The article "MicroRNA-34a regulates liver regeneration and the development of liver cancer in rats by targeting Notch signaling pathway" was retracted in 2024. Reasons: plagiarized images; overlap with other authors' work; concerns about the authorship; concerns about a third party's involvement.

# MicroRNA-34a regulates liver regeneration and the development of liver cancer in rats by targeting Notch signaling pathway

**DOI:** 10.18632/oncotarget.14807

**Published:** 2017-01-25

**Authors:** Xiao-Ping Wang, Jian Zhou, Ming Han, Chuan-Bao Chen, Yi-Tao Zheng, Xiao-Shun He, Xiao-Peng Yuan

**Affiliations:** ^1^ Third Division of Organ Transplant Center, The Eastern Hospital of The First Affiliated Hospital, Sun Yat-sen University, Guangzhou 510700, P. R. China

**Keywords:** microRNA-34a, liver regeneration, liver cancer, Notch signaling pathway

## Abstract

**Objective:**

This study aimed to investigate the role of microRNA-34a (miR-34a) in regulating liver regeneration (LR) and the development of liver cancer in rats by targeting Notch signaling pathway.

**Methods:**

Thirty male Sprague-Dawley (SD) rats were randomly assigned into partial hepatectomy (PH) group and sham hepatectomy (SH) group. Hematoxylin and eosin (HE) staining was used to observe the histological change in liver tissues. Enzyme-linked immunosorbent assay (ELISA) was used to measure the serum tumor necrosis factor α (TNF-α) and interleukin-6 (IL-6) levels. Dual-luciferase reporter gene assay was performed to examine whether miR-34a targeted Notch1 gene. Human liver cancer Huh7 cells were transfected and divided into blank, negative control (NC), miR-34a mimics and miR-34a inhibitors groups. MTT and flow cytometry were used to detect cell growth, and cell cycle and apoptosis, respectively. Quantitative real-time polymerase chain reaction (qRT-PCR) was applied detect to the expressions of miR-34a and Notch receptor mRNA. Western blotting was performed to detect the protein expressions of Notch receptors, P21, Bax, Bcl-2 and Bcl-xL. Tumor xenograft in nude mice was done to observe tumor formation in different groups.

**Results:**

Compared to the SH group, miR-34a expression in liver tissues in the PH group decreased first and then increased to the normal level during LR. In early stage of LR, the expressions of Notch receptors and miR-34a were negatively correlated. Compared to the blank and NC groups, the cell growth was inhibited, cell cycle was mainly arrested in the G2/M phase and cell apoptosis rate increased in the miR-34a mimics group. Moreover, the expressions of miR-34a, P21 and Bax were up-regulated, while the expressions of Notch receptors, and Bcl-2 and Bcl-xL were down-regulated in this group. Additionally, the tumor growth in the miR-34a mimics group was reduced. The miR-34a inhibitors group showed contrary tendencies.

**Conclusion:**

Our study demonstrates that miR-34a regulated LR and the development of liver cancer by inhibiting Notch signaling pathway.

## INTRODUCTION

Liver cancer is a type of tumor consisting of hepatic angiosarcoma, hepatocellular carcinoma (HCC) and cholangiocarcinoma, where HCC takes up over 80% in liver cancer patients [1]. Liver cancer was reported to be the second leading killer among cancers in the world, with a morbidity of 782,000 and a mortality of 746,000 by 2012, more than half of which occurred in China [2]. Liver regeneration (LR) commonly turns up when adult liver is damaged by surgery or poisoning, which could prevent further damage or inflammation to adjacent tissues [3]. Besides, LR is one of the most helpful theoretical bases for researches on tissue, organ and cell regeneration after partial hepatectomy (PH) [4]. This ability is major characterized by proliferation of various mature cells, such as hepatic stellate cells (HSCs) and hepatocytes [5]. MicroRNAs (miRs) refers to short noncoding RNAs with 22 nucleotides, which might perform vital functions in cellular events, including apoptosis, differentiation as well as cell cycle and human cancers, by regulating gene transcription [6]. In the present research, the function of miRs in liver cancer has been a leading project in disease biology areas, which is expected to benefit therapy.

MicroRNA-34a (miR-34a), belonging to miR family with high conservation, is encoded on human chromosome 1 and is considered as a suppressor in human malignancies through its regulation of target genes [7]. A previous study found that miR-34a mimic might be a novel target molecule for the treatment of liver cancer as it significantly suppressed tumor cell growth [8]. Notch signaling pathway is a highly conserved pathway which possesses four Notch receptors (Notch1 ~ 4) and five Notch ligands (Delta-like-1/3/4 and Jagged1/2) [9]. Some Notch proteins are expressed in regenerated liver, and Notch1 plays a considerable role in LR [10]. Overexpressed Notch1 was found to regulate cell apoptosis and cell cycle to inhibit HCC growth in tumor development [11]. Though miR-34a was proved to target Notch signaling pathway in multiple tumors, such as glioblastomas, breast cancer, cervical cancer and choriocarcinoma [9, 12, 13], the role of miR-34a interacting with Notch signaling pathway in liver cancer remains to be discussed, so this study would like to explore whether miR-34a affects LR and cancer development by targeting Notch signaling pathway.

## RESULTS

### Histological change in liver tissues

The liver tissues in the SH group had typical hepatic lobule structure, and the liver cells arranged orderly (Figure 1A). In the PH group, at 0.5 d, the liver cells arranged disorderly, the cell swelling was obvious, the cytoplasm was sparse, necrosis of liver cells occurred, the liver sinusoid showed non-convergent morphological changes and there was blood stasis (Figure 1B); at 1 d, an increase of inflammatory cells and fibroblasts which extended from the portal area and intertwined with each other was seen, and there were necrosis of liver cells and rich in blood vessels in liver tissues (Figure 1C); after 3 d, the swelling and thinning of liver cells were gradually alleviated (Figure 1D).

**Figure 1:** HE staining of liver tissues in the SH and PH groups during LR **Note: A**. HE staining of liver tissue in the SH group; **B**. HE staining of liver tissue in the PH group at 0.5 d; **C**. HE staining of liver tissue in the PH group at 1 d; **D**. HE staining of liver tissue in the PH group after 3d; HE, hematoxylin and eosin; SH, sham hepatectomy; PH, partial hepatectomy.

### Serum TNF-α and IL-6 levels during LR

As shown in Figure 2, the serum TNF-α and IL-6 levels were significantly higher in the PH group than in the SH group at all time points after 0.5 d (*P* < 0.05). At 0.5 d after hepatectomy, the serum TNF-α level in the PH group increased significantly. At this time, the serum concentration of TNF-α was about 2 times of that at the beginning, and the concentration began to decline since then. The serum concentration of IL-6 began to increase at 0.5 d after hepatectomy (*P* < 0.05) and reached the peak at 1 d, and then it decreased gradually. Compared with TNF-α, the high concentration of IL-6 lasted longer, showing a more stable concentration change.

**Figure 2:** Serum TNF-α and IL-6 levels in the SH and PH groups during LR **Note: A**. serum concentration of TNF-α in the SH and PH groups at 0 d, 0.5 d, 1 d, 3 d, 5 d and 7 d after PH; **B**. serum concentration of IL-6 in the SH and PH groups at 0 d, 0.5 d, 1 d, 3 d, 5 d and 7 d after PH; SH, sham hepatectomy; PH, partial hepatectomy.

### Expression of miR-34a during LR

The results of qRT-PCR were presented in Figure 3. The miR-34a expression at 0.5 d after PH decreased to half of the level at 0 d (*P* < 0.05), and it reached the lowest level at 1 d which was about a quarter of that in the SH group (*P* < 0.05). Hereafter, the expression of miR-34a in the PH group began to increase and reached the highest level at 5 d which was significantly higher than that in the SH group (*P* < 0.05). After that, it generally returned to almost the same level as the SH group. There was no significant change in the expression of miR-34a in the SH group.

**Figure 3:** Expression of miR-34a in the PH and SH groups during LR **Note:** *, *P* < 0.05 compared with the SH group; PH, partial hepatectomy; SH, sham-hepatectomy.

### Association between miR-34a and Notch receptors at the early stage of LR

According to qRT-PCR and Western blotting (Figure 4), it was found that from 0 d to 1 d after PH, the protein and mRNA expressions of Notch1, Notch 4 and Hes1 kept increasing, while the expression of miR-34a decreased to its lowest level at 1 d. Since 1 d, the mRNA and protein expressions of Notch4 started to decrease, and they dropped to the lowest level at 5 d, after which the expressions gradually increased to the level before liver resection. In general, the mRNA expression of Notch1 was negatively related to that of miR-34a, and the protein expression of Notch1 decreased from 1 d to 5 d and increased from 5 d to 7 d. As for the expression of Hes1, it presented two ascending tendencies: the first peak appeared 1 d, and the second at 5 d which was, however, a little lower than the first peak. Overall, the mRNA and protein expressions of Hes1 both remained relatively high. To conclude, at the early stage of LR, the expression of miR-34a was significantly in negative correlation with the expressions of Notch1, Notch4 and Hes1.

**Figure 4:** The expressions of miR-34a and Notch receptors in rats **Note: A**. the mRNA expressions of miR-34a and Notch receptors during LR; **B**. the protein expressions of Notch receptors during LR; Hes1, hairy and enhancer of split 1.

### miR-34a targeted Notch1

An online predicting software Target Scan was used to identify the target site on which Notch1 bound to miR-34a. Figure 5A shows the sequence of 3′-UTR where Notch1 mRNA bound to miR-34a. The liver cancer cell lines (Huh7) were transfected with miR-34a/Notch1-WT or miR-34a/Notch1-MT recombinant plasmids. It was found that miR-34a mimics exerted no significant influence on the luciferases activity of miR-34a/Notch1-MT plasmid (*P* > 0.05), but it led to 65% reduction in the luciferases activity of miR-34a/Notch1-WT plasmid (*P* < 0.05) (Figure 5B).

**Figure 5:** MiR-34a targeted Notch1 **Note: A**. the sequence of 3′-UTR where Notch1 mRNA bound to miR-34a; **B**. dual-luciferase reporter gene assay, which indicated that miR-34a mimics could inhibit the luciferases activity of miR-34a/Notch1-WT plasmid, while it had no effect on the luciferases activity of miR-34a/Notch1-MT; *, *P* < 0.05; WT, wild type ; MT, mutant type.

### Cell proliferation in the blank, NC, miR-34a mimics and miR-34a inhibitors groups

According to results of MTT (Figure 6), no statistical difference was shown in OD value at 24 h among the four groups (all *P* > 0.05). Also, there was no significant difference in cell proliferation at 24 h, 48 h and 72 h between the blank group and the NC group (all *P* > 0.05). At 48 h and 72 h, the growth of cells in the miR-34a mimics group were inhibited obviously, with its OD value being significant lower than those in the blank group and the NC group (both *P* < 0.05), while the growth of cells in the miR-34a inhibitors group was speeded up, with its OD value being statistically higher than those in the blank and NC groups (both *P* < 0.05).

**Figure 6:** Cell proliferation in the blank, NC, miR-34a mimics and miR-34a inhibitors groups **Note:** transfection of miR-34a mimics inhibited cells growth, while transfection of miR-34a inhibitors speeded up cells growth; *, *P* < 0.05 compared with the blank group and the NC group; NC, negative control.

### Cell cycle in the blank, NC, miR-34a mimics and miR-34a inhibitors groups

According to the results of PI staining (Figure 7), the proportions of cells in G1 phase in the blank, NC, miR-34a mimics and miR-34a inhibitors groups were (56.68 ± 2.23)%, (56.80 ± 2.33)%, (57.65 ± 2.04)% and (55.33 ± 2.19)%, respectively; the proportions of cells in S phase in the four groups were (26.06 ± 1.01)%, (26.97 ± 2.21)%, (15.63 ± 1.68)% and (34.72 ± 2.55)%, respectively; the proportions of cells in G2/M phase in the four groups were (17.26 ± 1.22)%, (16.23 ± 0.12)%, (26.72 ± 0.36)% and (9.95 ± 0.37)%, respectively. No statistical difference in cell cycle distribution was seen between the blank group and the NC group (*P* > 0.05). Compared with the blank group and the NC group, the miR-34a mimics group had increased percentage of cells in G2/M phase and decreased percentage of cells in S phase (both *P* < 0.05), indicating that the proliferation of liver cancer Huh7 cells was significantly inhibited. Compared with the blank group and the NC group, the miR-34a inhibitors group had decreased percentage of cells in G2/M phase and increased percentage of cells in S phase (both *P* < 0.05), suggesting increased number of liver cancer Huh7 cells in mitotic phases.

**Figure 7:** Cell cycle in the blank, NC, miR-34a mimics and miR-34a inhibitors groups detected by PI staining **Note: A**. cell cycle in each group detected by PI staining; **B**. histogram of cell cycle distribution in each group; *, *P* < 0.05 compared with the blank group and the NC group; NC, negative control; PI, propidium iodide.

### Cell apoptosis in the blank, NC, miR-34a mimics and miR-34a inhibitors groups

According to the results for Annexin V/PI staining (Figure 8), the apoptosis rates of cells in the blank, NC, miR-34a mimics and miR-34a inhibitors groups at 48 h after transfection were (1.89 ± 0.22) %, (1.91 ± 0.25) %, (18.31 ± 1.56) % and (0.91 ± 0.06) %, respectively. Compared with cells in the blank group and the NC group, the liver cancer Huh7 cells in the miR-34a inhibitors group had significantly lower apoptosis rate, while those in the miR-34a mimics group had significantly higher apoptosis rate (all *P* < 0.05).

**Figure 8:** Cell apoptosis in the blank, NC, miR-34a mimics and miR-34a inhibitors groups at 48 h after transfection detected using Annexin V/PI staining method **Note: A**. cell apoptosis in each group detected by flow cytometry; **B**. histogram analysis of the cell apoptosis rate in each group; *, *P* < 0.05 compared with the blank group and the NC group; NC, negative control; PI, propidium iodide.

### Expressions of miR-34a and Notch receptor mRNA in the blank, NC, miR-34a mimics and miR-34a inhibitors groups

According to the results of qRT-PCR (Figure 9), the liver cancer Huh7 cells in the miR-34a inhibitor group had decreased expression of miR-34a and increased mRNA expressions of Notch1, Notch4 and Hes1 in comparison to the blank group and the NC group (all *P* < 0.05), while the cells in the miR-34a mimics group had increased expression of miR-34a and decreased mRNA expressions of Notch, Notch4 and Hes1 when compared with the blank group and the NC group (all *P* < 0.05). However, there was no statistically significant difference in the expressions of miR-34a, and Notch1, Notch4 and Hes1 mRNA between the blank group and the NC group (all *P* > 0.05).

**Figure 9:** Expressions of miR-34a and Notch receptor mRNA in the blank, NC, miR-34a mimics and miR-34a inhibitors groups **Note: A**. histogram analysis of the expression of miR-34a in each group; **B**. histogram analysis of the mRNA expression of Notch1 in each group; **C**. histogram analysis of the mRNA expression of Notch4 in each group; **D**. histogram analysis of the mRNA expression of Hes1 in each group; *, *P* < 0.05 compared with the blank group and the NC group; NC, negative control; Hes1, hairy and enhancer of split 1.

### Expressions of Notch signaling pathway-related proteins and cell cycle and apoptosis-related proteins in the blank, NC, miR-34a mimics and miR-34a inhibitors groups

Western blotting (Figure 10) showed that at 48 h after transfection with miR-34a mimics, liver cancer Huh7 cells had down-regulated protein expressions of Notch signaling pathway-related Notch1, Notch4 and Hes1 and apoptosis-related Bcl-2 and Bcl-xL, but had up-regulated expressions of cell cycle-related P21 and apoptosis-related Bax when compared with the blank group and the NC group (all *P* < 0.05). In contrast, liver cancer Huh7 cells transfected with miR-34a inhibitors had increased protein expressions of Notch1, Notch4, Hes1, Bcl-2 and Bcl-xL but decreased expressions of P21 and Bax when compared with the blank group and the NC group (all *P* < 0.05). And there was no statistically significant difference in the expressions of all above proteins between the blank group and the NC group (*P* > 0.05).

**Figure 10:** Expressions of Notch signaling pathway-related proteins and cell cycle and apoptosis-related proteins in the blank, NC, miR-34a mimics and miR-34a inhibitors groups **Note: A**. expressions of Notch signaling pathway-related proteins detected by Western blotting; **B**. histogram analysis of the expression of Notch1, Notch4, Hes1 proteins; **C**. histogram analysis of the expression of P21, Bax, Bcl-2, Bcl-xL proteins; *, *P* < 0.05 compared with the blank group and the NC group; NC, negative control; Bax, Bcl2-associated X protein; Bcl-2, B-cell lymphoma 2; Bcl-xL, B-cell lymphoma-extra large.

### Growth of xenograft tumor in nude mice in the blank, NC, miR-34a mimics and miR-34a inhibitors groups

In the experiment of tumor formation in nude mice (Figure 11), liver cancer cells in the miR-34a mimics group had attenuated tumorigenicity, with reduced tumor volume and weight (0.430 ± 0.044 g) in nude mice, while those in the miR-34a inhibitors group had obviously heavier tumor (1.125 ± 0.151 g), which showed significant difference in comparison to the blank group (0.759 ± 0.103 g) and the NC group (0.795 ± 0.123 g) (all *P* < 0.05). The results suggested that miR-34a could inhibit tumorigenicity of liver cancer cells.

**Figure 11:** The growth of xenograft tumor in nude mice the blank, NC, miR-34a mimics and miR-34a inhibitors groups **Note: A**. subcutaneous tumor xenograft in nude mice; **B**. comparison of tumor volume among four groups; **C**. comparison of tumor weight among four groups; *, *P* < 0.05 compared with the blank group and the NC group; NC, negative control.

## DISCUSSION

The liver can remarkably regenerate itself when physical, nutritional, vascular, chemical, or virus-triggered liver injury occur [14]. LR, a highly orchestrated process, can be modulated by a variety of miRs [15]. For instance, miR-17~92 facilitated LR in an oestrogen-dependent manner [16], an increased expression of miR-34a led to inhibited hepatocyte proliferation during the late phase of LR [17], and miR-21 was upregulated in the early stage of LR, which targeted Pellino-1 to regulate NF-kappaB signaling [18]. As the mechanisms are largely unclear, analysis about miRs and related target genes may provide new understanding to liver disease [16]. In the present study, we mainly focused on the role of miR-34a in LR and the development of liver cancer by investigating its association with Notch signaling pathway. Our data indicated that miR-34a regulated LR and liver cancer development by targeting Notch signaling pathway.

In the study, the expression of miR-34a decreased at the beginning of LR and then gradually increased to normal level, indicating the involvement of miR-34a in LR. The miR-34a is widely known for anti-oncogenic activity in liver cancer, and the activation of miR-34a by the transcription factor p53 suggests its potential role in the modulation of hepatic cell behavior [19–21]. Deregulation of miR-34a occurs owing to altered p53 expression [22]. Therefore, that variation of p53 during LR is believed to contribute to the changing expression of miR-34a. In addition, elevated miR-34a in the late phase of LR can greatly repress the proliferation of rat hepatocytes by down-regulating INHBB and Met expression in regenerating livers [23], as the silencing of INHBB could greatly decelerate the growth of rat hepatocytes in LR and an increase in Met could cause impaired LR [23, 24]. It is why miR-34a was gradually up-regulated to normal level in our study.

Besides, it is found that over-expression of miR-34a led to reduced expression of Notch receptors (Notch1 and Notch4) and Notch target gene (Hes1), suggesting that miR-34a regulates Notch signaling pathway in a negative manner. Notch signaling pathway plays a vital role in cell development, such as proliferation and apoptosis, hence alterations in Notch signaling pathway are associated with pathologies in some tissues, including liver [25]. For example, the decrease of Notch1 expression could suppress HCC cell growth *in vitro* [26]. Additionally, the activation of Notch and Jagged signaling pathways contributes to the differentiation and growth of hepatocytes during LR after PH [27], which is reflected with the expression of Hes1, a target of Notch signaling pathway. Notch 1 is a direct target gene of miR-34a [28], as the dual-luciferase reporter assay verified that miR-34a bound to the 3′ UTR-binding sites of Notch 1 mRNA in the present study. In cervical cancer and choriocarcinoma, forced expression of miR-34a could inhibit Jagged1 and Notch1 expression, thereby causing a reduced invasion capacity of tumor cells [9]. Besides, miR-34a suppressed the proliferation and induced apoptosis of human glioma U87 cells by reducing the expression of target gene Notch1 [29]. The inactivation of Notch1 signaling pathway by miR-34a was also proved to attenuate the aggressiveness of prostate cancer [30]. This regulation was confirmed at the protein rather than mRNA level, which was consistent with previous finding that miRs were mainly involved in posttranscriptional gene regulation [29, 31]. In line with these studies, we found that in liver cancer Huh7 cells in the miR-34a mimics group, miR-34a expression significantly increased, while the expressions of Notch1, Notch4 and Hes-1 decreased when compared with the blank and NC groups. Unlike the other three Notch receptors, however, Notch4 is absent of detectable signaling ability, instead it inhibits ligand-induced Notch1 signaling through Notch4 extracellular domain when the two receptors are concurrently expressed in cells [32]. This may explain why the expressions of Notch4 and Notch1 were synchronized in liver tissues and cells.

Finally, it's demonstrated that the low expression of miR-34a in liver cancer Huh7 cells resulted in a larger proportion of cells in the S phase, facilitated cell proliferation and lower cell apoptosis rate, implying that miR-34a acts as a suppressor in liver cancer. The miR-34a induces cell-cycle arrest, apoptosis or senescence in cancer cells [33]. Bcl-2 family contains proteins either facilitating cell survival (Bcl-w, Bcl-2, Bcl-xL and others) or promoting cell death (Bak, Bad, Bax and others) [34]. As miR-34a can significantly down-regulate the expressions of Bcl-2, Bcl-w and Bcl-xL [35], and up-regulate the expressions of Bax and P21 [36], it can be concluded that the low expression of miR-34a could results in the inhibition of cell apoptosis, which is in consistent with our findings. The inactivation of apoptosis is central to cancer development, therefore low expression of miR-34a can results in the occurrence and progress of cancer [37]. Additionally, miR-34a could down-regulate expression of Notch1, hence low expression of miR-34a contributes to the development and progression of human malignancies through promotion of Notch1, including pancreatic cancer and prostate cancer [38–40]. Inactivation of miR-34a has been found in colorectal, urothelial, mammary, ovarian and renal cell carcinomas [41]. From these two aspects, it could be well concluded that miR-34a is an inhibitor in liver cancer.

In conclusion, the present study revealed that miR-34a could promote LR and suppress the development of liver cancer by inhibiting Notch signaling pathway. The findings provide a tantalizing hint that miR-34a might be a new therapeutic target for liver cancer. However, further studies are needed to test the effect of miR-34a on more hepatic cell types to further support our finding.

## MATERIALS AND METHODS

### Ethics statement

All animal experiments were approved by the Ethics Committee of the Eastern Hospital of the First Affiliated Hospital, Sun Yat-sen University.

### Study subjects

In this study, 30 specific pathogen free (SPF) male Sprague-Dawley (SD) rats purchased from Hunan SJA Laboratory Animal Co., Ltd (Hunan, China), at age of 8 weeks and weight of 200 g to 225 g, were selected. All rats were fed in SPF-class housing in the same condition, with 2 rats in each cage. Rearing condition: sterile fodder, free access to sterile water, 12 h light and dark cycle, 22°C ~ 26°C, and 37% to 42% humidity.

### Model establishment

Partial hepatectomy (PH) was performed using Higgins method [42, 43]. The 30 male SD rats were randomly assigned into PH group (0.5 d, 1 d, 3 d, 5 d and 7 d) in which rats underwent 70% PH, and sham hepatectomy (SH) group, with three rats in each group. Surgery was performed after one week of adaptive feeding. Rats need to be food fasted 12 h before surgery and liquid fasted 6 h before surgery. Then they were narcotized for 2 ~ 4 h by intraperitoneal injection with 10% chloral hydrate in the proportion of 300 mg/kg, fixed, unhaired, and disinfected with 75% ethyl alcohol. A 1.5 cm incision was made along the rat ventrimeson, and the liver was taken out with tweezers. Sterile surgical thread was used to ligature the root segment of liver to be cut off in order to alleviate postoperative bleeding. Next, the liver was cut off along the site of ligation (about 2 mm away), whose left lateral lobe and median lobe (right median lobe, left median lobe and gall bladder) were resected (around 70% weight of a whole liver). The rest part of liver was sent back to enterocoelia, followed by injection with 1 ml normal saline and suture. The operation in the SH group was the same as that in the PH group, except for hepatectomy. In case of damage to main blood vessels or surrounding tissues, the model was considered unsuccessful. Two hours after surgery, the animals woke up and were able to stand up. Six hours later, the animals started to eat again. The animals were continuously monitored, and the model establishment was successful if the animals could maintain normal activities. At certain time points after surgery (0.5 d, 1 d, 3 d, 5 d and 7 d), the rats in all groups were put to death, and the same part of their liver tissues were obtained for following experiments.

### Hematoxylin and eosin (HE) staining

The liver tissues obtained at different time points after PH (0.5 d, 1d, 3 d, 5 d and 7d) were fixed with 10% formaldehyde, embedded in paraffin, cut into 4 μm sections and stained with hematoxylin and eosin (HE). Steps for HE staining were as follows: the tissues were sliced up (0.5 h before sectioning, the wax block was placed in a -20°C freezer), and then the sections were baked at 70°C for 4 h, dewaxed, hydrated in distilled water, stained with hematoxylin (1 min), differentiated in hydrochloric acid alcohol, blued in ammonia water, counterstained with eosin (7 s), dehydrated with ethanol at different concentrations (75%, 90% and anhydrous ethanol), transparentized with xylene I and xylene II, and finally mounted in neutral gum. The liver tissue sections were observed under a microscope.

### Enzyme-linked immunosorbent assay (ELISA)

At certain time points after PH (0.5 d, 1 d, 3 d, 5 d and 7 d), 3 ml of venous blood from inferior vena cava was drawn and injected into coagulation-promoting tubes. After coagulation at room temperature, the blood was centrifuged at 3000 rpm for 5 min, and the supernatant was collected. The concentrations of TNF-α and IL-6 were measured according to the instructions of an ELISA kit (R & D Systems, Minneapolis, MN, USA). The absorbance value (A) of each well was measured at 450 nm of a multi-function microplate reader (BMG, Ortenberg, Germany). The expressions of tumor necrosis factor α (TNF-α) and interleukin-6 (IL-6) in each group was calculated and a standard curve was drawn based on the calculation.

### Quantitative real-time polymerase chain reaction (qRT-PCR)

Total RNA was isolated from tissues and culture cell using Trizol® (Invitrogen Inc., Carlsbad, CA, USA) according to the manufacturer's instruction. After the total RNA was dissolved in ultrapure water pretreated with diethylpyrocarbonate (DEPC), the optical density (OD) values at 260 nm and 280 nm were detected by ND-1000 ultraviolet-visible (UV-VIS) spectrophotometer (Nanodrop, America) to evaluate the quality of total RNA, followed by the adjustment of RNA concentration. Besides, according to the instruction of MBI Fermentas kit (Fermentas, America), the reverse transcription of RNA was performed on ice. Reaction condition: 70°C for 10 min, ice bath for 2 min, 42°C for 60 min and 70°C for 10 min. The cDNA was stored at a -80°C freezer. The reaction system for qRT-PCR was prepared following the instruction of kit (Fermentas, America). The primer sequences are shown in Table 1. The reaction condition was as follows: pre-denaturation at 95°C for 30 s, denaturation at 95°C for 10 s, annealing at 60°C for 20 s, extension at 70°C for 20 s, 40 cycles in total. The detection was done using Bio-Rad iQ5 qRT-PCR apparatus (Bio-Rad, Hercules, CA, America). U6 was used as the internal reference of miR-34a, and β-actin as the internal reference of rest target genes. The expressions of genes were calculated using relative quantitative measurement [44], where 2^-ΔΔCt^ represented relative expression of each target gene. Each experiment was repeated for 3 times.

**Table 1:** Primer sequences for qRT-PCR

Target gene	Primer sequence
miR-34a	F: 5′-GGGTGGCAGTGTCTTAGC-3′
	R: 5′-CAGTGCGTGTCGTGGAGT-3′
U6	F: 5′-AACGCTTCACGATTTGCGT-3′
	R: 5′-CTCGCTTCGGCAGCACA-3′
Notch1	F: 5′-GAGTCACCCCATGGCTAC-3′
	R: 5′-GTGGCTGCACCTGCTGGG-3′
Notch4	F: 5′-CACTGAGCCAAGGCATAGAC-3′
	R: 5′-ATCTCCACCTCACACCACTG-3′
Hes1	F: 5′-TCAACACGACACCGGACAAAC-3′
	R: 5′-GGTACTTCCCCAACACGCTCG-3′
β-actin	F: 5′-GGGAAATCGTGCGTGACATTTTG-3′
	R: 5′-TGTGTTGGCGTACAGGTCTTTG-3′

Abbreviations: qRT-PCR, quantitative real-time polymerase chain reaction; Hes1, hairy and enhancer of split 1; F, forward; R, reverse.

### Western blotting

The total protein specimens of liver tissues and cells were extracted and added into 1 × sodium dodecyl sulfate (SDS) loading buffer. A total of 20 μl loading buffer subjected to 12% polyacrylamide gel electrophoresis, transferred to membrane and blocked in decolorizing shaking table by Tris-Buffered Saline and Tween 20 (TBST) containing 5% bovine serum albumin (BSA) at room temperature for 1 h. Then the confining liquid was removed, the membrane was placed into a plastic groove, and antibodies at certain concentrations prepared with 5% BSA were added, including Notch1, Notch2, Notch4, hairy and enhancer of split 1 (Hes1), P21, Bcl2-associated X protein (Bax), B-cell lymphoma 2 (Bcl-2), B-cell lymphoma-extra large (Bcl-xL) and β-actin (Cell Signaling Technology, Inc., Beverly, MA, America). The impression surface was put on the front, and the membrane was stored at a 4°C freezer overnight. Next day, the membrane was washed by TBST for 3 times (10 min each time), incubated at 4°C for 4 ~ 6 h with the addition of diluted second antibody (Abcam Inc., Cambridge, UK), and finally washed by TBST again (3 × 15 min). Chemiluminescence reagent A and reagent B (Santa Cruz Biotech, Santa Cruz, USA) were mixed at a proportion of 1:1 and dropwise dripped on the nitrocellulose (NC) membrane. The protein bands were developed by developing solution. Relative OD analysis was performed in all Western blotting bands.

### Cell culture

Human liver cancer cell line Huh 7 (Cell bank of the Chinese academy of sciences, Shanghai, China) was cultured in dulbecco's modified eagle medium (DMEM) (Gibco, Invitrogen, Carlsbad, CA, USA) supplemented with 10% fetal bovine serum (FBS) (Hyclone, Logan, Utah, USA) in a 37°C incubator with 95% humidity and 5% CO_2_ (Thermo Scientific 8000, Thermo, America). The monolayer cells were adherent to wall. When these cells grew to 90% adherence, they were subcultured. Then the culture solution was aspirated, and cells were washed by phosphate buffer solution (PBS) for 2 times and digested by 0.25% trypsin (Gibco, Invitrogen, Carlsbad, CA, USA) When the cells turned round and intercellular space became larger, the trypsin was removed. Finally, the cells were separated by DMEM containing 10% FBS and were passaged with routine method.

### Dual-luciferase reporter gene assay

The target gene of miR-34a was analyzed using biological prediction website (microRNA.org) to predict the possible target gene and obtain the sequence of fragment containing action sites. The DNA of liver cancer cell line was extracted in strict accordance with the instruction of TIANamp Genomic DNA Kit (TIANGEN Biotech (Beijing) Co., Ltd., Beijing, China). Meanwhile, the sequences of Notch1-3′-untranslated region (UTR)-WT (wild-type Notch 3′UTR) and Notch1-3′-UTR-MT (mutant-type Notch1 3′UTR missing the binding site of miR-34a) were designed. After the construction of luciferase report vector, Huh 7 cells were transfected, and the luciferase activity was determined using a dual-luciferase reporter gene assay kit (Promega Corporation, Madison, WI, USA). The medium was removed at 48 h after transfection, and the cells were washed twice by PBS, followed by the addition of 100 μl Passive Lysis Buffer (PLB) into each well, 15 min gentle shaking at room temperature and collection of cell lysis buffer. The procedure was set as pre-reading for 2 s and reading for 10 s, and the amount of luciferase assay reagent II (LARII) and Stop & Glo^®^ Reagent was 100 μl each time. Prepared LARII and Stop & Glo^®^ Reagent was added into luminous tube or plate containing cell lysis buffer (20 μl each sample) which was then detected by a luminometer (Modulus™, Turner BioSystems, Sunnyvale, CA, USA).

### Cell transfection

Cells were divided into four groups: blank group (without any transfected sequence), NC group (transfected with negative control sequence 5′-UUCUCCGAACGUGUCACGUTT-3′), miR-34a mimics group (transfected with miR-34a mimics sequence 5′-ACCGUCACAGAAUCGACCAACA-3′), and miR-34a inhibitors group (transfected with miR-34a inhibitor sequence 5′-ACAACCAGCUAAGACACUGCCA-3′). All oligonucleotide sequences were synthesized by Sangon Biotech Co., Ltd. (Shanghai, China). Huh 7 cells in logarithmic phase of growth were inoculated into 6-well-plate. When the cells reached 30% to 50% confluence in complete medium without antibiotic, they were transfected according to the instruction of lipofectamin 2000 (Invitrogen Inc., Carlsbad, CA, USA). The siRNA plasmid (final concentration: 50 nM) and 5 μl lipofectamin 2000 were diluted by 250 μl serum-free Opti-MEM (Gibco, Invitrogen, Carlsbad, CA, USA) through even mixture, respectively, and were then incubated for 5 min at room temperature. The two diluted solutions were mixed gently, incubated for 20 min at room temperature, added into cell-contained well, and incubated at 37°C incubator with 5% CO_2_. After 6 to 8 h, the culture solution was changed, the complete medium was added and the cells were incubated for 24 to 48 h for following experiments.

### MTT assay

When the transfected cells reached about 80% confluence, these cells were washed twice by PBS and digested by 0.25% trypsin enzyme for the preparation of single-cell suspension. After cell counting, the cells were inoculated into 96-well plate (3 × 10^3^ ~ 6 × 10^3^ cells/well), with 200 μl suspension per well, totally 6 wells. After a period, 20 μl of 5 mg/ml MTT solution (Sigma-Aldrich Chemical Company, St Louis, MO, USA) was added into each well. After 4 h incubation inincubator, the culture solution was abandoned. Then 150 μl dimethylsulfoxide (DMSO) (Sigma, America) was added into each well, and the culture plate was lightly shaken for 10 min. The absorbance (OD value) of each well was detected at the wave length of 490 nm by an ELISA meter (Modulus™, Turner BioSystems, Sunnyvale, CA, USA) at 24 h, 48 h, and 72 h, respectively. The cell growth curve was drawn by using time as horizontal ordinate and OD value as longitudinal coordinate. Each experiment was repeated 3 times.

### Flow cytometry

Cell cycle detection was conducted following procedures as follows. At 48 h after transfection, cells were collected, washed by pre-cooled PBS solution for 3 times, and centrifuged, with the aspiration of supernatant. After cell concentration was adjusted to 1 × 10^5^ cells/ml, these cells were fixed by 1 ml of 75% ethyl alcohol, stored overnight at 4°C, and washed by PBS for 2 times, after which the supernatant was discarded. And then, 100 μl RNase A was added in the dark, 30 min water bath was performed at 37°C, and 400 μl propidium iodide (PI) (Sigma-Aldrich Chemical Company, St Louis, MO, USA) was supplemented for cell staining. After 30 min incubation at 4°C, FACSCanto II flow cytometry (BD Biosciences, America) was used to detect cell cycle by recording the red fluorescence at the wavelength of 488 nm. Each experiment was repeated 3 times.

Apoptosis rate was measured as the following steps. At 48 h after transfection, cells were collected using flow cytometry tube and centrifuged for 5 min at 1000 r/min, followed by the removal of supernatant. Then the cells were washed by cold PBS for 3 times and centrifuged, with supernatant aspirated. In accordance with the instruction of Annexin V-FITC apoptosis detection kit (Sigma-Aldrich Chemical Company, St Louis, MO, USA), 150 μl binding buffer and 5 μl Annexin-V-FITC were added into each tube and well-mixed by shaking, followed by 15 min incubation in the dark. Next, 150 μl binding buffer and 5 μl PI dye (Sigma-Aldrich Chemical Company, St Louis, MO, USA) were added into tube and well-mixed by shaking. Finally, flow cytometry was used to detect cell apoptosis. Each experiment was repeated 3 times.

### Tumor xenograft in nude mice

Well-conditioned Huh 7 cells were collected after 48 h of transfection, digested and resuspended into cell suspension, after which the cells were counted. A total of 100 μl cells at concentration of 3 × 10^7^ cells/ml was transferred into a sterile centrifuge tube. The cells were injected into three nude mice (Hunan SJA Laboratory Animal Co., Ltd., Changsha, China), with 4 injection sites in each rat and 3 × 10^6^ cells in each injection site. Transfected cells were subcutaneously injected through into both left and right sides of front and back paws of each mouse with 1 ml sterile syringe. Mice with injection on the left side of front paw, right side of front paw injection, left side of back paw and right side of back paw were divided into blank, NC, mimics and inhibitors groups, respectively. After cultivation, the mice were routinely fed. The tumor formation was observed every day. And every other day, the length (L) and width (W) of tumors were measured by vernier caliper. Tumor volume = (L × W^2^) × 0.5. After 2 weeks, mice were killed using cervical dislocation when the diameter of tumors was over 2 cm, after which tumors were stripped and photographed.

### Statistical analysis

All data were analyzed by SPSS 21.0 statistical software (IBM-SPSS Inc., Chicago, IL, USA), and measurement data were expressed as mean ± standard deviation (SD). Comparison among multiple groups was analyzed by one-way analysis of variance (ANOVA), while pairwise comparison in the same group was analyzed by *t-*test. The correlation analysis was done by Pearson analysis. *P* < 0.05 was considered to be statistically significant.
